This article has been retracted.

# Telemetry Data Compression Algorithm Using Balanced Recurrent Neural Network and Deep Learning

**DOI:** 10.1155/2022/4886586

**Published:** 2022-01-10

**Authors:** Parameshwaran Ramalingam, Abolfazl Mehbodniya, Julian L. Webber, Mohammad Shabaz, Lakshminarayanan Gopalakrishnan

**Affiliations:** ^1^Department of ECE, KPR Institute of Engineering and Technology, Arasur, Coimbatore 641048, Tamilnadu, India; ^2^Department of Electronics and Communication Engineering, Kuwait College of Science and Technology, Kuwait City, Kuwait; ^3^Graduate School of Engineering Science, Osaka University, Osaka, Japan; ^4^Arba Minch University, Arba Minch, Ethiopia; ^5^Department of Computer Science Engineering, Chandigarh University, Ajitgarh, Punjab, India; ^6^Department of ECE, National Institute of Technology, Tiruchirappalli, India

## Abstract

Telemetric information is great in size, requiring extra room and transmission time. There is a significant obstruction of storing or sending telemetric information. Lossless data compression (LDC) algorithms have evolved to process telemetric data effectively and efficiently with a high compression ratio and a short processing time. Telemetric information can be packed to control the extra room and association data transmission. In spite of the fact that different examinations on the pressure of telemetric information have been conducted, the idea of telemetric information makes pressure incredibly troublesome. The purpose of this study is to offer a subsampled and balanced recurrent neural lossless data compression (SB-RNLDC) approach for increasing the compression rate while decreasing the compression time. This is accomplished through the development of two models: one for subsampled averaged telemetry data preprocessing and another for BRN-LDC. Subsampling and averaging are conducted at the preprocessing stage using an adjustable sampling factor. A balanced compression interval (BCI) is used to encode the data depending on the probability measurement during the LDC stage. The aim of this research work is to compare differential compression techniques directly. The final output demonstrates that the balancing-based LDC can reduce compression time and finally improve dependability. The final experimental results show that the model proposed can enhance the computing capabilities in data compression compared to the existing methodologies.

## 1. Introduction

Aerospace telemetry is a procedure in which sensors connected to a data collection system collect data on the internal or external forces impacting a spacecraft. Data is collected and transmitted to a ground station via a communication link. Users receive comments following the ground station's analysis. Spacecraft's environmental properties, as well as its components, are monitored via aerospace telemetry systems. This enables fault analysis and data processing. Furthermore, because the amount of storage and bandwidth available for transmission is limited, data compression is required to improve transmission efficiency and reduce transmitter power consumption.

Data compression consists of lossy and lossless compression to eradicate redundant information from the original data. Only an estimate of the original data can be reconstructed using lossy compression. Lossless compression is a sort of data compression technology that allows for effective reconstruction of original data from compressed data. The data in the original file is more efficiently rewritten using lossless compression. Lossless compression is used to decrease a file's size and increase the compression rates with no loss of quality. For telemetry data, a variety of lossless compression techniques are now in use.

Recurrent neural network (RNN) is the cutting-edge method for time series data, and it is employed by Apple's Siri and Google's voice recognition. It is the first technique to recall its input thanks to its internal storage, making it ideal for machine learning issues involving sequential data. It is one of the algorithms that have enabled the incredible advances in reinforcement learning over the last several years. In this paper, we'll go over the fundamentals of how recursive neural networks function, as well as the major difficulties and even how to fix them.

In [1], the authors proposed a differential clustering (D-CLU) compression technique for lossless compression of real-time aeronautical telemetry data. Due to correlation, it was discovered that utilizing a differential compression model successfully enhanced compression performance. The introduction of differential compression, on the other hand, came with two large and nonnegligible drawbacks. These were the criteria for dependability and compression ratio. The clustering technique and coding were supposedly used in D-CLU to tackle these two difficulties. A one-pass clustering algorithm was employed during the clustering stage. Instead, Lempel–Ziv–Welch and run-length encoding were utilized for data encoding in the coding stage, depending on the clustering results. D-CLU not only decreased the error propagation range, but also improved reliability due to its improved compression performance. While it was stated that the error propagation range was reduced, thereby increasing the overall system's reliability, distortion measures were not analyzed. To fix this, this study begins with preprocessing the original telemetry data by subsampling and averaging it.

Typically, the compression algorithm grouped complete phrases into the same kind if their compositions were comparable. However, when certain node probability tables have specialized formulations, the inference results are also incorrect. To address the aforementioned concerns, a compression algorithm and a sequential inference method were developed, and an improved compression inference algorithm (ICIA) was designed in [2] and subsequently extended for multistate node applications with independent binary parent nodes. It was shown to be the best tool for analyzing complicated multistate satellite systems, with considerable advances in dependability analysis. The time it takes to compress complicated multistate satellite systems for analysis, on the other hand, has remained unsolved. To address this problem, this research looks at the time compression takes using BRNN as well as the dependability. Compression time is also enhanced by balancing the compression intervals.

The method of SB-RNLDC is proposed in this article for telemetric data, extending the method of [1,2] without the use of clustering. Additionally, redundant and undesirable data is discarded in order to isolate the most pertinent data for compression. The original samples are taken from the telemetry matrix. Additionally, we improve the compression rate by averaging subsampled data using a sampling cycle. To execute lossless compression on data, first we establish a probability measurement that produces identical distributions for each sample; then, we obtain a BCI to accomplish LDC and therefore lower the compression time. The following are some of the significant technological advancements made by this SB-RNLDC approach.

- The SB-RNLDC method is introduced for aerospace applications to increase compression rate while minimizing compression time. This contribution is made possible by the model of SATDP and the model of BRN-LDC.
- To increase compression rate, a methodology called SATDP is applied. Subsampling and sample averaging are novel techniques for removing noise and irrelevant data.
- The BRN-LDC model is used to improve compression performance while minimizing compression time. The novel probability measurement structure (PMS) and BCIS are used to reduce the computational complexity.

Section 2 discusses related works.  Section 3 goes into great detail about the BRN-LDC approach. The experimental circumstances and the telemetric dataset used are described in Section 4.  Section 5 discusses the performance analysis of the experimental results, and Section 6 concludes the paper.

## 2. Related Works

The current state of affairs presents a structure of required data mining procedure for solving issues in telemetry data including error detection, prediction, succinct summation, and visualization of large quantities, as well as assisting in understanding the geostationary overall health and detecting the signs of anomalies [3]. DC techniques were applied in accordance with the data's coding scheme, quality, data type, and intended use. The purpose, methodology, performance parameters, and various applications of DC techniques are discussed. The DC techniques developed reduced the size of data but did not address the issues. To improve the embedding capacity, an efficient lossless compression method was designed in [4]. The approach as developed did not take compression performance into account. Reference [5] described a LDC method for wireless sensor networks (WSNs) that makes use of multiple code options. The developed method enabled the compression and alteration of the source data information at a higher rate of speed. The computational complexity, on the other hand, was not reduced. This research work determines the use of ANN-based approach to detect the faults on raw data streaming that comes from the monitoring systems in order to minimize the need of engineer curated data streams for adapting in different devices. Reference [6] developed a lossless compression mechanism for home appliances based on hardware data compression. The serial interface with hardware acceleration was designed to sample infrared (IR) and very high-frequency signals. To reduce the size of oversampled data and conserve flash memory space, a hardware-based data compression mechanism was used. To minimize the size of the compressed data, a software-based compression mechanism was used. However, it was unable to store the data.

In [7], a two-step referential compression method based on K-means and K-nearest neighbors was developed. It reduced access time and enhanced data loading. However, since progress has been made in nearly all domains of activity, this has resulted in exponential expansion in real operation. Reference [8] proposed a neural network probability prediction approach with maximum entropy paired with an efficient Huffman encoding scheme to meet these types of jobs. As a result, transmission efficiency has improved. The capacity and energy efficiency of sensors are their two main drawbacks. To increase the energy efficiency of sensors with processing and storage, [9] presented a DCT based on a genetic algorithm. To achieve a high compression ratio, first-order static code (FOST) and sequence code (SDC) were used. This was believed to improve the processing time and computation process. Conventional compression methods are unable to achieve these needs, necessitating massive sensor data processing at a high compression rate and low energy cost. However, the compression time was not reduced. Reference [10] introduced a PMLZSS approach using a high-speed LDC algorithm that not only increased compression speed but also maintained the compression rate.

In [11], another low-overhead selection technique was developed using the prediction-based transformation. The developed technique selects the optimal compressor and reduces data storage and I/O time overheads but fails to improve compression quality. Reference [12] developed a novel tree-based ensemble approach based on Bregman divergence, ensuring a greater compression rate. In [13], a unique data inference compression mechanism using a probabilistic algorithm for identifying the most likely location and object positioning was reported for big volume data. Not only was great accuracy claimed to be achieved, but also efficiency was claimed to be kept by identifying and deleting superfluous information. However, there was no improvement to the compression ratio. Compression was used in [14] to eliminate forensically significant signs.

Another class of referential compression techniques was developed in [15] by incorporating local alignments for extended needs. This resulted in an increase in execution time due to the reduced memory use. However, it was not stated that redundant material would be removed. To solve this issue, [4] used lossless compression to accomplish a multilayer localized n-bit truncation. Without a doubt, LDC is quite prevalent. However, practically all LDC and decompression algorithms are shown to be extremely inefficient when parallelized, as they rely on sequentially updated dictionaries. The primary objective of [16] was to develop a novel LDC model called adaptive lossless (ALL) data compression. When utilized with graphics processing units (GPU), the model was constructed in such a way that the data compression ratio was reasonable, while decompression was efficient.

In [17], video compression algorithms that significantly reduce the size of the compressed video were developed. Although the designed methods achieved a better compression ratio, the image quality was degraded. Another lossless compression study for scientific datasets was conducted in [18] using a digital routing technique. To get a higher compression ratio, a digit rounding technique was included. The compression speed, on the other hand, was slower. Reference [19] examined the performance of data compression devices in depth, utilizing both quantitative rate-distortion analysis and subjective image quality evaluations. The image quality of the intended system was enhanced; however, the processing complexity was overlooked.

In [20], the authors proposed the PGF-RNN to develop lossless compression techniques. The gated recurrent units were altered to improve layer correlation in order to aggregate the fully linked layers and successfully locate the compressed data's features. To extract temporal features from compressed text data, an RNN-based architecture was used. Postprocessing was used to consider the frequency of bit sequences. The designed method enhanced the performance, but failed to apply the preprocessing approach. High-performance hardware architecture for both lossless and near-lossless compression modes of the LOCOI algorithm was introduced in [21] with higher throughput. The designed approach improved the compression ratio, and the complexity was not addressed.

In [22], the authors suggested a hardware-based DNN compression technique for addressing the memory constraints of edge devices. DNN weights were compressed using a novel entropy-based approach. For hardware implementation, a real-time decoding approach was used. The method devised enables the decompression of a single weight in a single clock cycle. The designed approach enhances the compression ratio. However, the compression time was not minimized. A novel highly efficient data structure was developed in [23] based on the premise that the matrix has a small number of shared weights per row. A sparse matrix data structure was used for decreasing the size and execution complexity. Not only were the designed data structures observed to be a generalization of sparse formats, they also provide more energy and time. However, they failed to eliminate redundant data.

In [24], the authors introduced an effective finite impulse response filter based on metaheuristic techniques, a game theory-based approach to improving image quality. Three blocks constitute the designed method: compression based on game theory, FIR filtering, and estimation of errors. The designed method eradicates the errors and noises, minimizing redundancy and improving the information in the original image. However, the computational complexity was not reduced. A new optimal approach named OSTS was presented in [25] for enhancing the segmentation of time series. Suboptimal methods for time series segmentation were used for attaining the pruning values. A suboptimal method that depended on the bottom-up technique was chosen. Then, the outcome of the suboptimal method was employed as pruning values for minimizing the computational time. However, it failed to reduce the computational complexity.

The vast majority of known research compresses data into blocks and processes them in parallel. However, it is claimed that data duplication occurs since compression is performed in parallel within the block. In the conventional works, preprocessing model is used to reduce the redundant and unwanted data. However, the compression performance was not addressed, and the minimization of computational complexity and compression time failed. The existing encoder and decoder were used to compress images for enhancing the image quality. However, the image quality needed to be improved. Additionally, because of the limited learning model used, the compression was not found to be optimal in real situations. Thus, the focus of our work is on reducing duplicate data in telemetric data via a considerable preprocessing model, as well as on neural network-based data compression methods and their applications to aerospace.

## 3. Methodology

The telemetric testing model is used to determine the aircraft's performance and to diagnose faults during flying tests by comparing the aircraft's responses to many input sensor signals. The testing signals are thought to serve two critical roles, transmission and storage. During transmission, testing signals are sent to the ground test station using the telemetry system's wireless media. In the event of storage, telemetry data or information is saved in a recorder, the contents of which are recycled following the experiment. Thus, an extremely effective communication channel transmission and telemetry data storage are critical due to the increasing quantity and variety of testing data, as well as the requirement for high real-time testing. Apart from telemetry, data compression increases the rate at which signal channels and storage capacity are used.

Telemetry data collected from multiple sensors on airplanes is in the form of text, pictures, audio, and video, among other formats with varying compositions. Only numerical data is considered in the suggested work, and a lossless compression approach is used. As a result, the telemetry data is converted to a digital format. However, the telemetry signals acquired by a telemetry system operating at a high sample rate include both competent and interfering signals. Thus, the signals must be preprocessed prior to performing LDC in order to mitigate the detrimental effect of noise on LDC. To accomplish this, a novel approach is proposed; it consists of two modularized phases: (1) preprocessing, subsampling, and averaging the telemetry data; (2) LDC using a BRNN model with an error parameter. The proposed method's architecture is depicted in Figure 1.

As seen in the figure, a typical SB-RNLDC model consists of two functional models: The subsampled averaged telemetry data preprocessing (SATDP) model preprocesses telemetric data by minimizing the dynamic range of errors and redundancy. Following that, a BRNN-LC model utilizes two structures to increase compression performance: a PMS and a BCIS. The following section contains a detailed description of the proposed method.

### 3.1. SATDP Model

The original telemetry data comprise measurements of several parameters obtained by multiple sensors, all sampled with the same sampling rate. Assume that “TM_*i*_={TM_*i*1_, TM_*i*2_,…,  TM_*ij*_,   …, TM_*in*_}” denotes the telemetry sample data acquired at a time “*t*,” where “TM_*ij*_” denotes the “*j* − *th*” data element. The original telemetry data is then represented by a telemetry matrix [1] “TM_(*a*∗*b*)_” and is expressed as follows:

(1) $$\begin{array}{c} {\text{TM}}_{a*b}=\left[\begin{array}{c} {\text{TM}}_{1}\\ \vdots \\ {\text{TM}}_{i}\\ \vdots \\ {\text{TM}}_{a} \end{array}\right]\left[\begin{array}{ccc} {\text{TM}}_{11} & {\text{TM}}_{1j} & {\text{TM}}_{1b}\\ \vdots & \vdots & \vdots \\ {\text{TM}}_{i1} & {\text{TM}}_{ij} & {\text{TM}}_{ib}\\ \vdots & \vdots & \vdots \\ {\text{TM}}_{a1} & {\text{TM}}_{aj} & {\text{TM}}_{ab} \end{array}\right]. \end{array}$$

The matrices (1), “*a*” and “*b*,” respectively, represent the number of samples and elements collected at each sampling instant. To mitigate noise's detrimental influence on LDC, the suggested method begins with preprocessing telemetry data using telemetry data in the form of a telemetry matrix. Prior to LDC, subsampling and averaging techniques are used for preprocessing. Subsampling eliminates redundant data and thus undesired data or noise. Adaptive sampling (AS) is used in this case to decrease telemetry traffic and storage by selecting events that are linked to the values of the variable of interest. This is mathematically expressed as follows:

(2) $$\begin{array}{c} {\text{TM}}_{\text{ss}}=\alpha {\text{TM}}_{\text{os}}. \end{array}$$

The telemetry matrix with subsampled data “TM_ss_” and the telemetry matrix with original samples “TM_os_” are produced using the adaptive sampling factor and the telemetry matrix with original samples “TM_os_,” respectively, from (2). Following that, the subsampled data are balanced using the following approach. To keep sample logic simple, four nodes, “*A*(*t*_0_), *A*(*t*_1_), *A*(*t*_2_), *A*(*t*_3_),” are sampled in a single sampling cycle. The four sample points are balanced using an average factor to minimize the detrimental influence of noise on LDC (i.e., the elimination of redundant data). After that, the averaged data “*A*(*T*_1_)” is written to the compression register. The subsampled averaged telemetry data preprocessing (SATDP) model is depicted in Figure 2.

As indicated in the SATDP model, the telemetry data is obtained in matrix form as input. Following that, subsampling of the telemetry data is undertaken. Subsampled data is supposed to reduce noise (i.e., redundant data) and hence eliminate useless data. Following that, averaging at different time intervals is conducted on the subsampled data to minimize the harmful effect on LDC. This procedure is repeated until all telemetry data associated with the related telemetry matrices has been processed. All averaged data are expressed in the following manner.

(3) $$\begin{array}{c} {\text{TM}}_{pq}=A\left(T_{1}\right),A\left(T_{2}\right)\text{,}\ldots ,A\left(T_{n}\right). \end{array}$$

The telemetric subsampled averaged data “TM_*pq*_” is obtained from (3) for the corresponding telemetry matrices, which are then compressed using lossless compression as discussed in the following section.

### 3.2. BRN-LDC Model

The BRN-LDC model is used to preprocess telemetry data with the goal of lowering memory requirements, station contact time, and data archival volume. The BRN-LDC model is said to ensure complete reconstruction of the original data without distortion. Additionally, by removing superfluous and redundant data from the aerospace application source data, the BRN-LDC model retains the correctness of the source telemetry data. On the other hand, during decompression, the compressed telemetry data is used to rebuild the original data by restoring the removed unneeded and redundant data. After the compression operation is complete, the resultant telemetry data structure is packetized in the format provided in Table 1.

The the lossless data packets are subsequently delivered through a packet data system from the source space ship to the data sink. These packets are then broadcast across the space-to-ground communication channel in such a way that the ground system can obtain the telemetric data with confidence. The package contents are then recovered and decoded from the underground sinks. The current work examines RNN and Kolmogorov complexity-based compressors, as well as the resulting BCI value, using preprocessed telemetry data. The suggested method achieves the BCI by employing Kolmogorov sophistication compressors. The BRN-LDC model is made up of two structures, that is, the PM and BCI architecture.

For a telemetric data stream “TM_*pq*_= TM_11_,  TM_*jk*_,…, TM_*pq*_,” the RNN PMS evaluates the probability distribution of “TM_*jk*_,” based on the previously observed samples “TM_os_= TM_11_,  TM_12_,   …, TM_*jk*−1_.” This probability measurement “Prob(TM_*jk*_*|*TM_11_,  M*T*_*jk*_,   …, TM_*pq*_)” is then fed into the BCI structure. At the end of the RNN estimator structure, there is a Softmax layer for estimating the probability measure. The RNN PMS takes as input only previously encoded symbols as features. This is expressed as follows:

(4) $$\begin{array}{c} \sigma \left(\text{TM}\right)pq=\;\frac{e^{{\text{TM}}_{p}}}{e^{{\text{TM}}_{q}}}. \end{array}$$

From (4), the exponential function “*e*(TM_*p*_)” is applied to each element “TM_*pq*_” of the input telemetric data vector “TM,” and these values are normalized by dividing the sum of all the exponentials in order to ensure that the sum of the components of the output vector (TM) equals to 1. Following that, the encoder and decoder weights are updated. This is critical, as both the encoder and decoder must yield comparable distributions for each symbol. The weight update is expressed in the following manner:

(5) $$\begin{array}{c} \Delta W_{pq}=\frac{\partial E_{\text{total}}\left(t_{0},t_{1}\right)}{\partial W_{pq}}. \end{array}$$

From (5), weights update “Δ*W*_*pq*_” is performed by applying the total cost function “*E*_total_” and sum overtime “*t*_0_, *t*_1_,…, ” of the standard error function to the partial derivatives “∂*W*_*pq*_” of multiple instances.

The BCI is a compression factor-based measure of similarity between two data files that approximates the Kolmogorov complexity. A novel compression algorithm for deep neural networks named DeepCABAC was introduced in [26]. It depended on using a context-based adaptive binary arithmetic coder (CABAC) for the parameters of the network. A novel quantization scheme was used in the DeepCABAC with reducing the rate-distortion function. The designed DeepCABAC improves the compression rate, but the neural network's issue was not solved. To address these difficulties, the BCI structure receives an estimate of the probability distribution for the following sample and encodes it as a state. This BCI permits the comparison of telemetry data packets from two data files while maintaining the lossless compression of the original files and avoiding the feature extraction approach often employed in compression and decompression. Finally, the decoder's operation is reversible. The BCI keeps a range of [0, 1], with each symbol stream setting its own range. This range is determined linearly and is reliant on the succeeding sample's probability estimate. This range is referred to as the BCI's state, and it is carried on for the following iterations. Finally, this range is encoded, resulting in the compressed data. Given the probability estimates, the decoding operations are inverse operations. The BCI is stated mathematically as follows:

(6) $$\begin{array}{c} {\text{BCI}}_{p,q}=\frac{C\left(p,q\right)-\text{MIN}\left\{c\left(p\right),C\left(q\right)\right\}}{\text{MAX}\left\{c\left(p\right),C\left(q\right)\right\}}. \end{array}$$

The BCI for the corresponding telemetry data in the form of matrices with “*p*” rows and “*q*” columns is calculated using the size of the compressed file obtained by the concatenation of “*C*(*p*, *q*),” with respect to the minimum concatenation “MIN*C*(*p*), *C*(*q*)” and the maximum concatenation “MAX*C*(*p*), *C*(*q*)”. The pseudocode representation of BRN-LDC is given below (Algorithm 1).

In the BRN-LDC approach described above, two procedures are performed. Initially, sub-sampling and averaging techniques are used to sample the telemetry data. Preprocessing of telemetric data sample is used to remove unnecessary and redundant features. A BRNN is used for LDC to increase the computational efficiency of preprocessed sample telemetric data. This is said to be done in this manner by combining derivative of a function with the BCI.

### 3.3. BRNED

Finally, this component performs encoder and decoder operations.  Figure 3 illustrates the BRNED operations. The BCI begins with a default estimate of the probability distribution for the first sample “S0.” This is done so that the decoder can decode the first sample.

DeepZip, lossless compressor using recurrent networks, was introduced in [26] for enhancing lossless compression. The designed method was faster but did not work well on more complex sources. In order to overcome this issue, BRNED operations are introduced. As illustrated in Figure 3, both the BCI and PMS retain state information between iterations. The BCI's final state serves as lossless compressed data.

## 4. Experimental Settings

The proposed BRNN-LDC algorithm's performance is tested in this part via numerical simulation using MATLAB. The suggested SB-RNLDC method uses a predictive maintenance telemetry dataset that includes data from a variety of sources, including telemetry, failures, maintenance, errors, and machines.

The first dataset is telemetry time series data, which is made up of real-time vibration voltage, rotation, and pressure measurements taken by 100 machines and averaged each hour in 2015. The second data source is the error logs, which contain nonbreaking faults that do not result in machine failures. Due to the hourly acquisition of telemetry data, the incorrect dates and times are also rounded to the nearest hour. Scheduled and unplanned maintenance records, which pertain to both routine component inspections and component failures, are the third data source. When a component is replaced during a scheduled inspection owing to a failure, a record is created or replaced. The fourth data source is machines, which represent the model type and year of service. Finally, the final data source keeps track of component failures and component replacements. The compression rate, compression time, and computational complexity of the SB-RNLDC approach are all measured and compared to two current methods, D-CLU [1] and ICIA [2].

## 5. Results and Discussion

The SB-RNLDC approach is compared to two state-of-the-art methods in this section, namely, D-CLU [1] and ICIA techniques [2].

### 5.1. Performance Estimation of Compression Rate

The data compression rate is used to quantify the size reduction in the data representation produced by the balanced RNN data compression method. To put it another way, the compression rate is used to assess the algorithm's efficiency. As a result, compression rate is defined as the size of uncompressed data divided by the amount of compressed data.

(7) $$\begin{array}{c} \text{CR}=\frac{U_{\text{Size}}}{C_{\text{Size}}}. \end{array}$$

The compression rate (CR) is determined by comparing the size of the uncompressed telemetric data length “*U*_Size_” to the size of the compressed telemetric data length “*C*_Size_” in (7). A value closer to zero indicates improved compression, while a value more than one indicates negative compression; i.e., the compressed image size is greater than the reference image size. Below are sample compression rate calculations for the proposed SB-RNLDC method, as well as the existing algorithms, namely, D-CLU and ICIA.

#### 5.1.1. Sample Computation

(i) Proposed algorithm SB-RNLDC: the overall compression rate is presented below using 15 samples as input, the length of telemetric data before compression is 175, and the length of telemetric data after compression is 125.
  (8) $$\begin{array}{c} \text{CR}=\;\frac{175}{125}=1.4. \end{array}$$
(ii) Existing algorithm D-CLU: consider 15 telemetric samples taken as input, the length of telemetric data before compression is 175, and the length of telemetric data after compression is 135; an overall compression rate is as follows:
  (9) $$\begin{array}{c} \text{CR}=\;\frac{175}{135}=1.2963. \end{array}$$
(iii) Existing algorithm ICIA: consider 15 telemetric samples taken as input, the length of telemetric data before compression is 175, and the length of telemetric data after compression is 145; an overall compression rate is provided below.

(10) $$\begin{array}{c} \text{CR}=\;\frac{175}{145}=1.2069. \end{array}$$

Figure 4 shows the compression rates for a variety of samples utilizing the novel SB-RNLDC method as well as the established D-CLU algorithm [1] and ICIA method [2]. In the majority of samples, it can be shown that the SB-RNLDC approach performs better than the other two methods. To enable a fair comparison of the three methods, simulation parameters range from 15 to 150. SB-RNLDC technique outperforms D-CLU algorithm [1] and ICIA method [2], but D-CLU algorithm [1] outperforms ICIA methodology [2]. The SB-RNLDC technique, for instance, compresses all samples to near-zero levels, implying that the compressed data volume exceeds the uncompressed data volume. This is because the SB-RNLDC approach employs Kolmogorov complexity-based compressors to determine the BCI. Compression performance is supposed to be enhanced through the acquisition of the BCI. This enhancement is supposed to increase the compression rate of the SB-RNLDC approach by 10% when compared to D-CLU algorithm [1]. Furthermore, because only finite data sequences are relevant in probability applications, the BCI combined with the Kolmogorov complexity with the shortest description avoids redundant data in the telemetric matrix, increasing the compression rate of the SB-RNLDC method by 27 percent over ICIA [2].

### 5.2. Performance Estimation of Compression Time

A LDC technique's CT value should be as small as possible. Due to the bigger amount of the telemetric data, the CT of the telemetric data is fairly high in comparison to conventional data.

(11) $$\begin{array}{c} \text{CT}=\text{samples}*\text{time}\left(\text{compression}\right). \end{array}$$

Compression time is calculated using the sample size and time consumed during compression in (11). Milliseconds are used to quantify it (ms). The suggested SB-RNLDC approach, as well as the existing D-CLU and ICIA methods, has a sample compression time calculation.

#### 5.2.1. Sample Computation

(i) Proposed SB-RNLDC: with a total of 15 samples selected for testing and a compression time of 0.035 ms for a single sample, the total compression time is as follows:
  (12) $$\begin{array}{c} \text{CT}=15*0.035\text{ ms}=0.525\text{ ms.} \end{array}$$
(ii) Existing D-CLU: with a total of 15 samples selected for testing and a compression time of 0.043 ms for a single sample, the total compression time is as follows:
  (13) $$\begin{array}{c} \text{CT}=15*0.043\text{ ms}=0.645\text{ ms.} \end{array}$$
(iii) Existing ICIA: with a total of 15 samples selected for testing and a compression time of 0.051 ms for a single sample, the total compression time is calculated as follows:

(14) $$\begin{array}{c} \text{CT}=15*0.051\text{ ms}=0.765\text{ ms.} \end{array}$$

The compression time for 150 different samples is compared in Figure 5. Figure 5 plots each compression time interval across 150 distinct samples. The figure shows that the compression time increases as the number of samples increases. For instance, when 15 distinct samples were considered, the time required to compress them into a single sample was found to be 0.035 ms using the SB-RNLDC method, 0.043 ms using D-CLU algorithm, and 0.051 ms using ICIA method. Thus, the overall compression time was determined to be 0.525 ms, 0.645 ms, and 0.765 ms, respectively, utilizing the SB-RNLDC, D-CLU algorithm, and ICIA methods. As a result, the sample size is proportional to the compression time, as shown in the diagram. The overall amount of data increases as the number of samples increases, and so does the time necessary to compress it. However, the proposed SB-RNLDC approach should result in a faster compression time. This is because two distinct procedures are utilized, namely, subsampling and sample averaging. Subsampling was proven to be effective in reducing irrelevant data. This resulted in a 22 percent reduction in compression time when compared to D-CLU when employing the SB-RNLDC approach [2]. Apart from the application of averaging to balance the subsampling points, the SB-RNLDC approach was shown to lower compression time by 33 percent when compared to ICIA method [2].

### 5.3. Performance Estimation of Computational Complexity

The term “computational complexity” refers to the amount of memory required to compress and decompress data. The method's efficiency is assured by its low computational complexity. It is expressed in the following way:

(15) $$\begin{array}{c} \text{CC}=\text{samples}*\text{MEM}\left(\text{compression}\right). \end{array}$$

As demonstrated in (15), the computational complexity (CC) is dictated by the size of the telemetry matrix containing original samples “Samples” and the amount of memory spent during compression. It is quantified in kilobits (KB). The new SB-RNLDC approach has been compared with the current D-CLU and ICIA methods in terms of computational complexity.

#### 5.3.1. Sample Computation

(i) Proposed SB-RNLDC: with a total of 15 samples and a single sample consuming 12 KB of memory during compression, the overall computational complexity is as follows:
  (16) $$\begin{array}{c} \text{CC}=15*12\text{ KB}=180\text{ KB.} \end{array}$$
(ii) Existing D-CLU: with 15 samples taken into account and a single sample consuming 18 KB of memory during compression, the overall computational complexity is as follows:
  (17) $$\begin{array}{c} \text{CC}=15*18\text{ KB}=270\text{ KB}. \end{array}$$
(iii) Existing ICIA: with 15 samples taken into account and a single sample consuming 23 KB of memory during compression, the overall computational complexity is as follows:

(18) $$\begin{array}{c} \text{CC}=15*23\text{ KB}=345\text{ KB.} \end{array}$$

Figure 6 depicts the convergence plot of computational complexity for samples evaluated in the range of 15 to 150 samples at various time intervals. The quantity of memory used by the LDC process is referred to as computational complexity. The difficulty of computation is reported to be varied depending on the number of samples acquired from telemetric data for experimentation. Reduced computing complexity ensures the method's efficiency. Furthermore, as seen in the diagram, the number of samples is proportional to the computational complexity. This is because the existence of extraneous material in telemetric data that is not deleted during preprocessing has a detrimental influence on the complexity rate. However, the BRN-LDC is supposed to reduce computational complexity while maintaining a high rate of reliability and a short compression time. Additionally, the computational complexity is reduced as a result of these enhancements. To begin, redundant data is practically eliminated when both subsampling and averaging are used, resulting in a higher compression rate. Compression time is stated to be lowered with an increased compression rate. By SB-RNLDC approach, computational complexity is stated to be lowered by 15% compared to [1] and 23% compared to [2].

## 6. Conclusion

The intricate nature of telemetric data with high dimensional characteristics degrades overall efficiency during data compression. This article describes the SB-RNLDC method. The fundamental contribution of this study is to increase the compression rate of the data produced by the SATDP model. Telemetry data was collected from various time periods. The sample telemetric data was then subsampled and balanced using average parameters to increase the compression rate. The subsampled and balanced telemetric data were then put into the BRN-LDC model to speed up compression. Finally, it was revealed that the PM and BCI may be employed to reduce computation complexity. When compared to earlier attempts, MATLAB experiments show that the proposed technique is more efficient in terms of compression rate, compression time, and computing complexity. According to the results, the Kolmogorov complexity-based compressors achieve a greater compression rate, 28 percent of minimal compression time by using subsampling and averaging of the samples, and 19% less computational complexity with the aid of BRN-LDC model than the state-of-the-art methods.

The proposed model can be implemented in various practical applications where large amount of data needs to be handled. Some of its practical applications involve aerospace application, stock market, large data storing warehouses, and data transmission.

## Figures and Tables

**Figure 1:** The proposed SB-RNLDC technique architecture.

**Figure 2:** SATDP model.

**Figure 3:** BRNED.

**Figure 4:** Comparing compression rates for proposed SB-RNLDC and existing algorithms (D-CLU and ICIA).

**Figure 5:** Comparison of compression time for proposed SB-RNLDC and existing algorithms (D-CLU and ICIA).

**Figure 6:** Comparing of computational complexity for proposed SB-RNLDC and existing algorithms (D-CLU and ICIA).

**Algorithm 1:** Algorithm 1 BRN-LDC.

**Table 1:** Test telemetric data information as a packet.

S. No.	Date, time	Machine ID	Volt	Rotate	Pressure	Vibration
1	2015-01-01 06:00:00	1	176.217853015625	418.504078221616	113.077935462083	45.0876857639276
2	2015-01-01 07:00:00	1	162.87922289706	402.747489565395	95.4605253823187	43.4139726834815
3	2015-01-01 08:00:00	1	170.989902405567	527.349825452291	75.2379048586662	34.1788471214451
4	2015-01-01 09:00:00	1	162.462833264092	346.149335043074	109.248561276504	41.1221440884256
5	2015-01-01 10:00:00	1	157.61002119306	435.376873016938	111.886648210168	25.9905109982024

## Data Availability

The data shall be made available on request.
